# Acute Toxicity and Gastroprotection Studies of a New Schiff Base Derived Copper (II) Complex against Ethanol-Induced Acute Gastric Lesions in Rats

**DOI:** 10.1371/journal.pone.0051537

**Published:** 2012-12-10

**Authors:** Maryam Hajrezaie, Shahram Golbabapour, Pouya Hassandarvish, Nura Suleiman Gwaram, A. Hamid A. Hadi, Hapipah Mohd Ali, Nazia Majid, Mahmood Ameen Abdulla

**Affiliations:** 1 Department of Molecular Medicine, Faculty of Medicine, University of Malaya, Kuala Lumpur, Malaysia; 2 Department of Chemistry, University of Malaya, Kuala Lumpur, Malaysia; 3 Institute of Biological Science, Faculty of Science, University of Malaya, Kuala Lumpur, Malaysia; Center for Cancer Research, National Cancer Institute, United States of America

## Abstract

**Background:**

Copper is an essential element in various metabolisms. The investigation was carried out to evaluate acute gastroprotective effects of the Copper (II) complex against ethanol-induced superficial hemorrhagic mucosal lesions in rats.

**Methodology/Principal Findings:**

Rats were divided into 7 groups. Groups 1 and 2 were orally administered with Tween 20 (10% v/v). Group 3 was orally administered with 20 mg/kg omeprazole (10% Tween 20). Groups 4–7 received 10, 20, 40, and 80 mg/kg of the complex (10% Tween 20), respectively. Tween 20 (10% v/v) was given orally to group 1 and absolute ethanol was given orally to groups 2–7, respectively. Rats were sacrificed after 1 h. Group 2 exhibited severe superficial hemorrhagic mucosal lesions. Gastric wall mucus was significantly preserved by the pre-treatment complex. The results showed a significant increase in glutathione (GSH), superoxide dismutase (SOD), nitric oxide (NO), and Prostaglandin E2 (PGE_2_) activities and a decrease in malondialdehyde (MDA) level. Histology showed marked reduction of hemorrhagic mucosal lesions in groups 4–7. Immunohistochemical staining showed up-regulation of Hsp70 and down-regulation of Bax proteins. PAS staining of groups 4–7 showed intense stain uptake of gastric mucosa. The acute toxicity revealed the non-toxic nature of the compound.

**Conclusions/Significance:**

The gastroprotective effect of the Copper (II) complex may possibly be due to preservation of gastric wall mucus; increase in PGE_2_ synthesis; GSH, SOD, and NO up-regulation of Hsp70 protein; decrease in MDA level; and down-regulation of Bax protein.

## Introduction

Ulcer is an open sore or lesion, usually found on the skin or mucous membrane of the body. A peptic ulcer is a lesion occurs at the lining of the stomach or duodenum, where hydrochloric acid and pepsin are present. In the past, it was thought that lifestyle factors, such as stress and diet caused ulcers. Later, researchers found that stomach acids (i.e., hydrochloric acid) and pepsin took part in ulcer formation. Many researches have shown that most ulcers (80% of gastric ulcers and 90% of duodenal ulcers) contribute significantly to bacterium *Helicobacter pylori*. Among the three factors (lifestyle, hydrochloric acid and pepsin, and *H. Pylori*) important in ulcer development, *H. pylori* is the primary cause of the gastric ulcer [1], [2]. Stress is an important etiological factor in the incidence of gastric ulcer. Free radicals, in stress-involved gastrointestinal injuries, may inactivate synthetize of mucosal prostaglandin (by accumulating H_2_O_2_, an inhibitor in synthesis of the prostaglandin, which propitiates the generation of reactive oxygen species [3]. Lipid-derived free radicals such as conjugated dienes and lipid hydroperoxides cause oxidative reactions. The process of lipid peroxidation is mediated by the interaction between hydroxyl radicals and the cell membrane, during which the lipid-derived free radicals produce [4]. Recently, a numerous researches have been inclined to find effective synthetic chemical compounds with gastroprotective properties [5], [6], [7].

**Figure 1:** Chemical structure of Cu(BrHAP)_2_.

Copper is an essential trace element in human metabolism, but does not exist in ionic form in biological systems. The amount of copper in the body is measured in complexes with organic compounds. The process of chelating metals smuggles them to bypass the intestinal wall and to enter into the mainstream of nutrient flow and usage in the body. Copper complexes such as copper aspirinate and copper tryptophanate, remarkably increase healing rate of ulcers and wounds [8]. The Copper complexes shorten the healing period of gastric ulcers for five days and promote the wound healing process at the same time retaining anti-inflammatory activity [8] while non-steroidal anti-inflammatory drugs (e.g. ibuprofen and enefenamic acid) suppress wound healing process.In recent years, copper coordination compounds with schiff-base ligands have been extensively studied.It seems that their reactivity with dioxygen or its reduced derivativesistheirunique biological property [9]. Some of schiff base derived copper compounds causesevere cytotoxicity, through the generation of reactive oxygen species which can damage different biomolecules [10]. However, they may be considered as efficient catalyst for the oxidation of different substrates [11]. Many of these complexes have been investigated for their effective scavengers of superoxide radicals [12], acting as antioxidants.This study introduced the Copper (II) complex derived from N,N’dimethyl ethylene diamine and 2-hydroxyacetophenone schiff base ligand, its synthesis and its chemical characterization. Also, the study evaluated acute toxicity and gastroprotective activity of the complex against absolute ethanol-induced acute hemorrhagic mucosal lesions in rats.

**Table 1:** Elemental analysis and spectral characterization for the ligand and its metal complex.

Ligand	Elemental Analysis	Analytical Calculated: C, 69.87; H, 8.80; N, 13.58.
		Found: C, 68.48; H, 8.98; N, 14.98.
	IR (KBr disc cm−1)	υ(Ar–OH), 3436sb; υ(C–H), 2836s; υ(C = N), 1628s; υ(C–C), 1438s; υ(C–N), 1166s;
	UV-Vis (DMSO), λmax (ε, Mol−1cm−1):	279 nm (3091.79, π-π*); 303 nm (3152.21, CT)
	1H-NMR (DMSO-d6)	2.23 (s, 3H, CH3), 2.28 (6H, 2CH3), 2.49 (t, 2H, 2CH2), 6.78–7.02 (4H, ArH), 10.7 (s, 1H, phenolic)
	13C-NMR (DMSO-d6)	16.72 (CH3), 45.54 (2CH3), 45.86, 57.53 (2CH2), 167.91 (C = N) ArC: [125.15 (CH), 128.48(CH), 141.33 (CH), 1148.29 (CH), 149.82 (C)]
Complex	Elemental Analysis	Analytical Calculated: C, 40.29; H, 5.07; N, 7.83
		Found: C, 40.88; H, 5.20; N, 7.23.
	IR (ATR cm−1)	2843.53 m,2800.66 m ν(C-H), 1102.37 m ν(C-N), 1474.35 m, 1436.35 m ν(C-C), 1605.47 m, 1593.89 ν(C = N), 518.09 m ν(M-N), 473.95ν(M-O).
	UV-Vis (DMSO)	296 (π→π*); 362 (n→π*); 376 (LMCT); 610 (d→d*).

## Materials and Methods

### Experimental Section

All of the chemicals used in this study were obtained from Fluka and Aldrich and used as received without further purification. Schiff bases were synthesized by condensation reaction. The two ethanolic solutions were stirred for 2 h or 5 h after dissolving it. The ethanol was then evaporated using Rota evaporator. Infrared spectra were obtained using KBr discs (4000–400 cm^−1^) on Perkin –Elmer FT-IR spectrometer. Elemental analysis (C, H, N) were performed using a Flash EA 1112 Series elemental analyzer in University of Technology Malaysia.

### Synthesis of the Copper Complex

2-hydroxyacetophenone (0.21 g, 1.65 mM) was weighed accurately and was dissolved in 25 mL of absolute ethanol dripping to an ethanolic solution and N,N′dimethylethyldiamine (0.14 g, 1.65 mM) at room temperature and was refluxed for 3 h. A clear yellow oily product was formed after the evaporation process. The product was isolated in liquid form by adding a few drops of diethyl ether/n-hexane and the purity was confirmed by TLC. Stoichiometric amount of the synthesized schiff base ligand (1.65 mM) was dissolved in 25 mL absolute ethanol, an equimolar quantity of Copper (I) bromide (0.21 g, 1.65 mM) in a minimum amount of ethanol was added. A blue precipitate was formed. The precipitate was filtered, washed with ethanol and dried in vacuum desiccators. Recrystallization was performed in ethanol. The crystal structure of the compound X-ray [13] is as shown in the proposed structure in Figure 1. Elemental analysis and spectral characterization for the ligand and its metal complex are presented in the Table 1.

**Figure 2:** Histological sections in acute toxicity test (H & E staining, 20x). Histological sections of liver (first row) and kidney (second row) in acute toxicity test. Rats treated with 5 mL/kg vehicle (10% Tween 20) (A and D). Rats treated with 500 mg/kg (5 mL/kg) the Copper (II) complex (B and E). Rats treated with 2000 g/kg (5 mL/kg) the Copper (II) complex (C and F). There is no significant differences in structures of liver and kidney between treated and control groups.

**Figure 3:** Macroscopical appearance of the gastric mucosa in rats. The negative control group (A) has no injury of gastric mucosa. The ulcer control group (B) shows sever injuries in the gastric mucosa. Absolute ethanol produced extensive visible hemorrhagic necrosis of gastric mucosa. The reference control group (omeprazole, 20 mg/kg) (C) shows mild injuries in the gastric mucosa comparing to the injuries seen in group 2. Rats received 10 mg/kg of the complex (D) has moderate injuries in the gastric mucosa. The extract reduces the formation of gastric lesions induced by absolute ethanol. Rats received 20 mg/kg of the complex (E) shows mild injuries in the gastric mucosa. Rats received 40 mg/kg of the complex (F) shows mild injuries in the gastric mucosa. Rats received 80 mg/kg of the complex (G) does not show any injuries of the gastric mucosa instead flattening of gastric mucosa is visible (white arrow). Black arrows point to the superficial hemorrhagic mucosal lesions.

**Figure 4:** Effects of the complex on gastric ulcer area, inhibition percentage and alcian blue binding capacity. Alcian blue binding capacity is defined as Gastric wall mucus (GWM). Groups 1 to 3 represent the negative control group, the ulcer control group and the reference control group (omeprazole, 20 mg/kg), respectively. The experimental groups received 10, 20, 40 and 80 mg/kg of the complex are presented as groups 4–7, respectively. All values are expressed as mean ± standard error mean. Mean difference is significant, in GWM, at the *p*<0.05 level (one-way between groups ANOVA with post-hoc analysis). * significant when compared with the group 2. # significant when compared with the group 3. Inhibition of gastric lesions (%) is indicated in brackets above the columns.

**Figure 5:** Effect of the complex on glutathione (GSH), superoxide dismutase (SOD) and nitric oxide (NO) (A,B and C). Groups 1 to 3 represent the negative control group, the ulcer control group and the reference control group (omeprazole, 20 mg/kg), respectively. The experimental groups received 10, 20, 40 and 80 mg/kg of the complex are presented as groups 4–7, respectively. All values are expressed as mean ± standard error mean. Mean difference is significant at the *p*<0.05 level (one-way between groups ANOVA with post-hoc analysis). * significant when compared with the group 2. # significant when compared with the group 3.

**Figure 6:** Effects of the complex on malondialdehyde (MDA), prostaglandin E2 (PGE_2_) and protein concentration (A, B and C). Groups 1 to 3 represent the negative control group, the ulcer control group and the reference control group (omeprazole, 20 mg/kg), respectively. The experimental groups received 10, 20, 40 and 80 mg/kg of the complex are presented as groups 4–7, respectively. All values are expressed as mean ± standard error mean. Mean difference is significant at the *p*<0.05 level (one-way between groups ANOVA with post-hoc analysis). * significant when compared with the group 2. # significant when compared with the group 3.

**Figure 7:** Histological study of gastric mucosal damage in rats (20x). In the negative control group 1 (A), no disruption to the surface epithelium is observed. The ulcer control group (B) has severe disruption to the surface epithelium (black arrows) and necrotic lesions penetrate deeply into mucosa and extensive edema of submucosal layer (yellow arrows) and leucocyte infiltration (blue arrows) are present. The reference control group (omeprazole, 20 mg/kg) (C), mild disruption of the surface epithelium mucosa is present but deep mucosal damage is absent. Reduction of submucosal edema and leucocytes infiltration is seen. Rats received 10 mg/kg of the complex (D) has moderate disruption of surface epithelium with submucosal edema and leucocytes infiltration of submucosal layer. Rats received 20 mg/kg of the complex (E) shows mild to moderate disruption of surface epithelium. In rats received 40 mg/kg of the complex (F), there is mild disruption to the surface epithelium. Reduction of submucosal edema and leucocytes infiltration of the submucosal layer are shown. Rats received 80 mg/kg of the complex (G) has no disruption to the surface epithelium.

### Chemicals

In this study, omeprazole (obtained from UMMC Pharmacy) was used as the reference anti-ulcer medicine. The medicine was dissolved in 10% Tween 20 (Merck Schuchardt OHG, 85662 Hohenbrunn, Germany). A dilution of (10% v/v) Tween 20 was used as the vehicle for dosing all of the rats (5 mL/kg) and were administered orally to the rats in a dosage of 20 mg/kg body weight (5 mL/kg) according to the recommendation of Mahmood *et al.* [14].

### Experimental Animals

#### Acute toxicity study

Healthy male and female Sprague-Dawley rats (6–8 weeks old) were obtained from the Animal House, Faculty of Medicine, University of Malaya, Kuala Lumpur (Ethics No. PM/27/07/2010/MAA (R). The rats were weighed between 150–180 g. The animals were given standard rat pellets and tap water ad libitum. The acute toxicity study was used to determine a safe dose for the Copper (II) complex. 36 rats (18 males and 18 females) were randomly assigned into 3 groups labeled as vehicle (10% Tween 20), and 100 mg/kg and 2000 mg/kg of the Copper (II) complex (10% Tween 20) [15]. The animals were fasted overnight prior to the dosing. Food was withheld for another 3 to 4 h after dosing. The animals were under observation for 0.5, 2, 4, 8, 24 and 48 h after administration to monitor any onset of clinical or toxicological symptoms. Mortality, if any, was recorded over a period of 2 weeks. The animals were sacrificed on day 15. Histology, hematological and serum biochemical parameters were determined according to the OECD [15]. This study was approved by the Ethics Committee for animal experimentation, Faculty of Medicine, University of Malaya, Malaysia Ethic No. PM/07/05/2011/MAA (R). Throughout experiments, all of the animals received humane care according to the “Guide for the Care and Use of Laboratory Animals” prepared by the National Academy of Sciences.

**Figure 8:** Effect of the complex on gastric tissue glycoprotein-PAS staining (20x). The negative control group (A), the ulcer control group (B), the reference group (omeprazole, 20 mg/kg) (C), rats received 10 mg/kg of the complex (D), rats received 20 mg/kg of the complex (E), rats received 40 mg/kg of the complex (F), and rats received 80 mg/kg of the complex (G). Magenta color in the apical epithelial cells in the treated groups with the compound (groups 4–6) shows gradual increase in mucosal secretion of gastric glands. The intense secretion of mucus in gastric glands is demonstrated in group 7. The arrow points to the glycoprotein accumulation.

**Figure 9:** Immunohistochemical analysis of expression of Hsp70 proteins (20x). The negative control group (A), the ulcer control group (B), the reference group (omeprazole, 20 mg/kg) (C), rats received 10 mg/kg of the complex (D), rats received 20 mg/kg of the complex (E), rats received 40 mg/kg of the complex (F), and rats received 80 mg/kg of the complex (G). Immunohistochemistry staining of Hsp70 shows over-expression of Hsp70 protein in the experimental groups (D-G). The arrow points to the Hsp70 protein accumulation.

**Figure 10:** Immunohistochemical analysis of expression of Bax proteins (20x). The negative control group (A), the ulcer control group (B), the reference group (omeprazole, 20 mg/kg) (C), rats received 10 mg/kg of the complex (D), rats received 20 mg/kg of the complex (E), rats received 40 mg/kg of the complex (F), and rats received 80 mg/kg of the complex (G). Immunohistochemistry staining of Bax proteins shows down-expression of Bax protein in D-G. The arrow points to the Bax protein accumulation.

#### Gastric ulcer study

Sprague Dawley healthy adult male rats were obtained from Experimental Animal House, Faculty of Medicine, University of Malaya; Ethic No. PM/28/09/2011/MAA (R). The rats (weighed between 225–250 g) were divided randomly into 7 groups consisting of 6 rats each group. Each rat was caged individually with wide-mesh wired bottoms to prevent coprophagia during the experiment. The animals were maintained on a standard pellet diet and tap water ad libitum.

#### Gastric ulcer-induced by ethanol

Prior to the experiment, the rats were fasted for 24 h, according to a recommended method [14]. They had free access to drinking water till 2 h before the experiment. Gastric ulcer was induced by orogastric intubation of absolute ethanol (5 mL/kg) according to the method recommended by Abdulla *et al.* [14]. Group 1 and group 2 were orally administered with 10% Tween 20 (5 mL/kg). Group 3 received an oral dose of 20 mg/kg omeprazole in 10% Tween 20 (5 mL/kg), as the reference control group. The experimental groups were orally administered with the Copper (II) complex dissolved in 10% Tween 20 (5 mL/kg) at different dosages of 10, 20, 40 and 80 mg/kg (Groups 4, 5, 6 and 7, respectively). Then, 1 h after this pre-treatment, group 1 was orally administered with 5 mL/kg 10% of Tween 20.Groups 2–7 were received absolute ethanol orally (5 mL/kg). The rats were euthanized 60 min later (based on the previously used method [16]) with an overdose of xylazine and ketamine anesthesia and their stomachs were immediately excised.

#### Macroscopic appearance of acute gastric mucosal lesion

Lesions of the gastric mucosa appear as elongated bands of superficial hemorrhagic mucosal lesions parallel to the long axis of the stomach. Gastric mucosa of each rat was thus examined for the damages. The length and width of the hemorrhagic mucosal lesions (mm) were measured with a planimeter (10 × 10 mm^2^ = ulcer area) under a dissecting microscope (1.8x). The hemorrhagic mucosal lesions area was measured by counting the number of small squares (2 mm × 2 mm) covering the length and the width of each lesion band. The sum of the areas of the lesions for each stomach was applied in a calculation of the UA where the sum of small squares × 4 × 1.8 = UA (mm^2^) were calculated according to the recommendation of Zahra *et al.* [17]. The inhibition percentage (I%) was calculated by the following formula according to the recommendation of Abdulla *et al.* [18].


#### Gastric wall mucus determination

The glandular segments of the stomach were removed, weighed and assessed to determine gastric wall mucus in rats [19]. Each segment was transferred immediately to a 1% alcian blue solution (in sucrose solution, buffered with sodium acetate at pH 5).Rinsing with sucrose solution, the excess dye was removed. The dye complexed with the gastric wall mucus was extracted by magnesium chloride solution. A 4 mL aliquot of blue extract was then shaken with an equal volume of diethyl ether. The resulting emulsion was centrifuged then the absorbance of the aqueous layer was measured at 580 nm. The quantity of alcian blue extracted per gram of glandular tissue was then calculated.

#### Preparation of stomach homogenate

The gastric tissue homogenate from each rat was prepared for PGE2 and MDA assays. The entire experiment was performed at 4°C. Gastric tissue was cut into 3 small pieces (approximately 200 mg for each), and the exact weight of each piece was recorded [20]. The tissues were homogenized in a teflon homogenizer (Polytron, Heidolph RZR 1, Germany) using the appropriate buffer. The amount of buffer used was dependent on the weight of the tissue used. After centrifugation at 4,500 rpm for 15 min at 4°C, the supernatant was used for the PGE2 and MDA assays.

#### Antioxidant activities of stomach homogenate

The GSH levels of the gastric tissues were measured using gastric tissue supernatant with the GSH kit (Cayman Chemical Co., Mich, USA), according to the manufacturer’s instructions. The SOD activities in the gastric tissues were determined, according to the manufacturer’s protocol, using the SOD assay kit (Cayman Chemical Co., Mich, USA). Using a commercial kit (Cayman Chemical Co., Mich, USA), the NO levels of gastric tissues were measured according to the manufacturer’s instructions.

### Enzymatic Activities of Stomach Homogenate

#### Measurement of membrane lipids peroxidation (MDA)

The rate of lipoperoxidation in the gastric mucous membrane is valued through the measurement of MDA using the TBARS test. The stomachs were washed with normal saline to minimize any interference of hemoglobin with free radicals and to remove blood adhered to the mucous membrane. The stomachs were homogenized with potassium phosphate buffer (10% (w/v). A total of 250 µL was then stored at 37°C for 1 h. Then 400 µL of 35% perchloric acid was added. The mixture was centrifuged at 14,000 rpm for 20 min at 4°C. The supernatant was mixed with 400 µL of 0.6% thiobarbituric acid and incubated at 95–100°C for 1 h. After cooling, the absorbance was measured at 532 nm. A standard curve was used for the calculation by 1,1,3,3-tetrametoxypropane. The results were expressed nM of MDA/mg of protein. The concentration of the proteins was measured using the method described by Bradford assay [21]. The measurement of total protein in the stomach sample is based on the interaction between the Coomassie Blue G250 dye and proteins. The interaction of high molecular weight proteins with the dye causes a shift in the ionic charge of the dye to the anionic form, with strong absorbance at 595 nm. To run the assay, a proper volume of albumin standard, distilled water, buffer solution and each sample were added to the wells. For a sample preparation, 2 µL of a sample and 38 µL of the buffer solution were added to a well. Then, 200 µL Bradford's solutions (diluted 5×) were added to the well. After 5 min, the absorbance was recorded at the wavelength of 595 nm [21].

#### Measurement of PGE2 formation

The gastric mucosa was weighed, minced with scissors, and homogenized at 4°C in PBS buffer, accordingly. Homogenates were centrifuged at 13 400 g for 10 min. The supernatants were subjected to a PGE2 assay using a PGE2 Monoclonal Enzyme Immunoassay Kit (Sigma-Aldrich, Malaysia).

#### Measurement of protein concentration

Protein concentrations (mg/ml tissue) were determined using the Biuret reaction, as described by Gornall et al. [22].

### Histological Evaluation of the Gastric Lesions

#### Hematoxylin and eosin staining technique

Specimens of the gastric tissue were fixed in 10% buffered formalin and were processed in the paraffin tissue-processing machine (Leica, Germany). Sections of the stomach were sectioned at 5 µm and stained with hematoxylin and eosin for histological evaluation [23].

#### Study of mucosal glycoproteins

Sections of the glandular portion of the rat stomach of each group were stained with PAS stain to observe mucus production and to evaluate changes in both acidic and basic glycoproteins [24].

#### Immunohistochemical evaluation

Slides of the tissue sections heated at 60°C for 25 min in a hot-air oven (Venticell, MMM, Einrichtungen, Germany). The tissue sections were de-paraffinized in xylene and were rehydrated using graded alcohol. Antigen retrieval process was performed in 10 mM sodium citrate buffer boiled in microwave. Immunohistochemical staining was conducted according to manufacturer's protocol (Dakocytomation, USA). Briefly, endogenous peroxidase was blocked by peroxidase block (0.03% hydrogen peroxide containing sodium azide). The tissue sections were washed gently with the washing buffer. Then the sections were incubated with Hsp70 (1∶500) or Bax (1∶200) biotinylated primary antibodies for 15 min. The sections were rinsed gently with wash buffer and place in the buffer bath. The slides were then placed in a humidified chamber. Sufficient amount of streptavidin–HRP (streptavidin conjugated to horseradish peroxidase in PBS containing an anti-microbial agent) was incubated with the sections for 15 min. Then, the tissue sections were rinsed gently in the washing buffer and were place in the buffer bath. DAB-substrate-chromagen was incubated with the sections for 5 min, following washing and counterstaining with hematoxylin for 5 sec. The sections were then dipped in weak ammonia (0.037 M/L) 10 times and were rinsed with distilled water prior to the mounting of cover slips. Positive findings of the immunohistochemical staining are shown in brown color under a light microscope.

### Statistical Analysis

All of the values were reported as mean ± SEM. The statistical significant differences between groups were assessed using one-way ANOVA. A value of *p*<0.05 was considered significant.

## Results

### Acute Toxicity Study

In the acute toxicity study, the animals were treated with the Copper (II) complex at a dosage of 100 mg/kg and 2000 mg/kg and were kept under observation for 14days. All of the animals were alive and did not manifest any sign of toxicity at these dosages. There was no detectable sign of hepatic or renal toxicity in the treated groups as compared with the control group (Figure 2 and Table S1).

### Macroscopic Evaluation of Gastric Lesions

Gross comparison of the stomachs among the groups is illustrated in Figure 3.The results showed that rats in the groups 4–7 had significantly reduced areas of gastric mucosal lesions formation compared to rats in group 2 (*p*<0.05). The Copper (II) complex significantly suppressed the formation of the hemorrhagic mucosal lesions and interestingly flattened the gastric mucosal folds in group 7 (Figure 3G). Furthermore, absolute ethanol-induced mucosal lesions were significantly reduced in term of size and severity among the rats received the pre-treatment of the Copper (II) complex. The gastroprotective activity of the Copper (II) complex in the ethanol-induced acute hemorrhagic mucosal lesions model is shown in Figure 4. The inhibition of hemorrhagic mucosal lesions in groups 4–7 was remarkable in comparison with the group 3 (Figure 3 and Figure 4).

### Gastric Wall Mucosal Evaluation

Gastric wall mucus was significantly reduced in the group 2. Rats pre-treated with the Copper (II) complex showed meaningful inhibition of the depletion of gastric wall mucus. In the group 2, the gastric wall mucosal was significantly decreased following the ethanol administration. But, the pre-treatment with the Copper (II) compound significantly inhibited this reduction (Figure 4).

### Antioxidant Activities of Stomach Homogenate

Rats in the group 2 showed significant reductions in the levels of GSH, SOD and NO as compared to those in the group 1, whilst, rats in the groups 3–7 showed compensatory increases (Figures 5).

### Biochemical Assays of MDA and PGE_2_ in Gastric Tissue Homogenate

Administration of absolute alcohol significantly surged the MDA level of the gastric homogenate in comparison to group 1. The MDA level of the gastric tissue in the groups 3–7 was decreased as compared with group 2 (Figure 6A). In the gastric mucosa homogenate, the level of PGE_2_ was decreased in group 2(compared to the group 1). Groups 3–7 showed increases in the PGE_2_levels as compared to group 2 (Figure 6B). These results indicated that pre-treated with the complex increased the level of PGE_2_ in the tissue homogenate as shown in the groups 4–7, demonstrating the possible protective property of the compound against acute hemorrhagic mucosal lesions (Figure 6B). Protein concentration in gastric homogenate was significantly decreased in the group 2 compared with the group 1. Administration of the complex significantly increase the protein content of gastric homogenate compared with the group 1 (Figure 6C).

### Histological Evaluation of Gastric Lesions

Histological observation of the ethanol-induced gastric mucosal lesions in group 2, showed comparatively extensive damage to the gastric mucosa, and edema and leukocytes infiltration of the submucosal layer (Figure 7). Rats received pre-treatment with the Copper (II) complex showed comparatively better protection of the gastric mucosa by reduction in ulcer area, edema and leukocyte infiltration of the submucosal layer (Figure 7).

### Periodic Acid Schiff (PAS) of Mucosal Glycoproteins

Increased in the level of PAS staining of gastric mucosa in groups 4–7 in comparison to group 2 indicated the increase in the glycoprotein content of the gastric mucosa. Group 4–7 reversed the decrease in PAS staining induced by ethanol as shown in Figure 8.

### Immunohistochemistry

Immunohistochemical results showed that rats in the groups 4–7 had over-expression of Hsp70 protein (Figure 9). The expression of Hsp70 protein in group 2 was down-regulated as compared to the group 4–7 (Figure 9). Immunohistochemical staining of Bax protein demonstrated that rats in the groups 4–7 had down-expression of Bax protein (Figure 10). Ethanol, as shown in the group 2, up-regulated the expression of Bax, whilst pre-treatment with the complex decreased the expression of this protein in the groups 4–7 by (Figure 10).

## Discussion

The IR spectra of the complex possesses very strong characteristic absorption bands in the region of 1585–1656 cm^−1^ attributed to the C = N stretching vibration of the schiff base imino functional group [25], [26]. The spectra for the complex show M–N bands at a lower wavelength in the range of 454–556 cm^−1^ [7], [27].

The electronic spectra for the complex is obtained in DMSO solvent and showed absorption bands in three-distinct regions. The first region, ranging from 221 to approximately 229 nm, is characteristic for the electronic inter ligand π→π* transitions [28], while the second characteristic wavelength, in the region of 281 nm to approximately 322 nm, is the second inter ligand n→π transition [29]. The third distinct region, ranging from 407 nm to approximately 498 nm, is the characteristic for the LMCT from the nitrogen atom to the transition metal center [30].

Acute toxicity test did not show any signs of toxicity and mortality over a period of 14daysand emphasized on that the Copper (II) complex was safe to be used. No hepatic toxicity and no renal toxicity were seen through the biochemistry and histology results. Ethanol-induced gastric mucosal lesions made it possible to evaluate gastroprotective activity [31]. Ethanol is metabolized in the body and releases superoxide anions and hydroperoxy free radicals. Oxygen-derived free radicals are implicated in the mechanism of acute and chronic ulceration in the stomach [32]. The genesis of ethanol-induced gastric lesions showed a multifactorial origin with a decrease in gastric mucus, and was associated with the significant production of free radicals, leading to increased lipid peroxidation which in turn caused damage to cells and cell membranes [33]. The results of the present study showed that the Copper (II) complex possessed an effective anti-ulcer activity against ethanol-induced hemorrhagic mucosal lesions in rats. The compound increased the gastric wall mucus, inconsistent with the results previously reported by Salga *et al.* [6]. The gastroprotective effect of the compound appeared to be mediated partly through the preservation of gastric mucus secretion.

Omeprazole, a proton pump inhibitor, offered a fairly protected gastric mucosa has been widely used as an acid inhibitor agent in treatment of disorders related to gastric acid secretion [34]. Omeprazole, besides its anti-secretory effect, and effectiveness in acid-dependent ulcer models, is effective in acid independent models, like ethanol-ulcer model, and exert mucosal protection in non-anti-secretory doses [35].

Changes in gastric motility is important in development and prevention of experimental gastric lesions [18]. In the present study, the flattening of the mucosal folds suggested that the gastroprotective effect of the compound was due to decrease in gastric motility. The Flattening of the folds increased the mucosal area exposed to the necrotizing agents, and reduced the volume of the gastric irritants on rugal crest [16], [18].

Increase in the level of GSH appeared consistent with the adaptation phenomenon, the higher the GSH level, the less the damage occurred. GSH and other antioxidants prevented tissue damage by keeping reactive oxygen species at their physiological levels [36]. SOD is able to convert superoxide to hydrogen peroxide, and subsequently, the catalase converts hydrogen peroxide to water. Reduction in the activity of SOD was observed in the gastric mucosa homogenate in the ulcerated rats. This is likely that SOD is utilized in the decomposition of superoxide anion generated by lipid peroxidation. The decrease in the activity of SOD in the hemorrhagic lesions might be resulted from a number of deleterious effects. Pre-treatment with the Copper (II) complex increased the activity of SOD which suggested this effect as a gastroprotective method of the complex in reduction of lipid peroxidation. On the contrary, previous study showed that the activity of SOD increased in the ethanol treated group compared to the normal rats [37]. The Copper (II) complex maintained the level of SOD similar to the normal control group. It seemed that the Copper (II) complex could decrease the oxidative stress condition caused by ethanol.

Ethanol effectively reduced the level of nitric oxide NO in the gastric mucosa and slowed the flow of gastric blood, thereby caused the development of hemorrhagic lesions and consequently led to solubilisation of gastric mucus constituents. These actions resulted in an increased flow of Na+ and K+, an increase in pepsin secretion, loss of H+ ions and histamine into the lumen [38], [39]. NO had the ability of inhibiting the neutrophil infiltration to provide a protective barrier for the gastric mucosa against ethanol [40]. The Copper (II) complex enhanced the production activity of NO. Similarly, synthesis of NO protected the gastric mucosa against damage induced by various ulcerogenic models [41]. This finding introduced the ability of the Copper (II) complex to increase the level of NO content as a gastroprotective agent.

As mentioned before, oxidative damage is an important reason for cell membrane damage. MDA is the final product of lipid peroxidation and is used to determine lipid peroxidation levels [42]. Our results showed that gastric tissue homogenate in the pre-treated rats with the Copper (II) complex exhibited significant antioxidant activity by decreasing the levels of MDA and by elevating the levels of PGE_2_ in response to oxidative stress. Lipid peroxidation is known as important pathophysiological event in a variety of diseases [43]. So, the level of MDA is a biomarker for oxidative stress [44]. PGE_2_ is crucial in the regulation of gastric mucus secretion. PGE_2_showed protective effects against various gastric injury models [45]. Ethanol is able to reduce the mucosal PGE_2_ content [46]. PGE_2_asthe most abundant gastrointestinal prostaglandin, regulates functions of the gut, including motility and secretion [47]. PGE_2_exerts a protective action on the stomach through the activation of E prostanoid receptors [48]. Cytoprotection by prostaglandin is unrelated to the inhibition of gastric acid secretion since prostaglandin increases the resistance of gastric mucosal cells to the necrotizing effect of strong irritants. Prostaglandins maintain the cellular integrity of the gastric mucosa, and maybe beneficial in the treatment of a variety of diseases in which gastric mucosal injury is present [46]. The results of the current study reveal that protection against gastric mucosa lesions and inhibition of leucocytes infiltration into the gastric wall happened in the rats pre-treated with the Copper (II) complex. Group 2 showed that activation and infiltration of neutrophils, initiate the formation of the lesion. Similarly, Abdulla *et al.* reported that the reduction of neutrophil infiltration into ulcerated gastric tissue enhanced the prevention of gastric ulcers in rats [18]. Absolute alcohol extensively damages the gastric mucosa, leading to increased neutrophil infiltration into the gastric mucosa. Neutrophils mediate lipid peroxidation through the production of superoxide anions [49]. Neutrophils are the major source for inflammatory mediators and can release potent reactive oxygen species such as superoxide, hydrogen peroxide and myeloperoxidase derived oxidants.

This study showed that mucosal level of PGE_2_ was significantly enhanced by the Copper (II) complex. The enhancement indicated a gastroprotective effect of the Copper (II) complex. Prostaglandins influence virtually every component stimulating mucus and bicarbonate secretion, maintaining mucosal blood flow, enhancing the resistance of epithelial cells to injury induced by cytotoxins and inhibiting leukocyte recruitment [50].

There is a variety of factors influence gastric ulcer prevention. For instance, mucus and bicarbonate secretion seems important in the ulcer preventing process because the mucus/bicarbonate layer protects newly formed cells from acid and peptic injury [51]. PAS staining exhibits characteristic carmine staining of stomach regions that secrete mucopolysaccharides. Group 7 showed intense secretion of mucus in gastric glands. Mucus production is one of the main mechanisms of local gastric mucosal defense [52].

Hsp70 proteins defend cells from oxidative stress or heat shock. Ethanol generates reactive oxygen species (ROS) which normally inhibits the expression of Hsp70 and enhances the expression of Bax. Hsp70 prevents these partially-denatured proteins from aggregating, and allows them to refold. Hsp70 is a 70 kDa protein from the Hsp family present on mammalian cells. It is the most conserved and abundantly produced protein in response to different forms of stress [53], such as heat, toxic agents, infection and proliferation [54]. These proteins are responsible to protect cellular homeostatic processes from environmental and physiologic injuries by preserving the structure of normal proteins and repairing or removing damaged proteins. Over-expression of Hsp70 proteins and down-regulation of Bax proteins were shown in this study that suggest these regulations a gastroprotective method of the Copper (II) complex against ethanol-induced superficial hemorrhagic mucosal lesions in rats.

### Conclusions

The Copper (II) complex derived from N,N’dimethyl ethylene diamine and 2-hydroxyacetophenone schiff base ligand did not cause any sing of acute toxicity in rats (100 mg or 2000 mg/kg). The compound could significantly protect the gastric mucosa against ethanol-induced injury. Antioxidant activities of GSH, SOD and NO were significant increase in the gastric mucosal homogenate, while there was a remarkable decrease in MDA. Assay of PGE_2_in the gastric tissue homogenates revealed significant increase in the PGE_2_ level in the pre-treated group with the complex as compared with the group 2. Such protection was ascertained grossly by significant increase in the gastric wall mucus in comparison with the ulcer control group. Also the reduction of hemorrhagic mucosal areas in the gastric wall as well as the reduction or inhibition of edema and leukocytes infiltration of the submucosal layers were shown histologically. Immunohistochemistry staining of Hsp70 and Bax proteins showed up-regulation of Hsp70 protein and down-regulation of Bax protein in rats pre-treated with the Copper (II) complex. Increased the PAS staining of gastric mucosa of treated animals in comparison to group 2 indicated the increase in glycoprotein content and the Copper (II) complex reversed the decrease in PAS staining induced by ethanol. This study provided histological evidences on gastroprotective property of the Copper (II) complex and suggested that the complex preserved of gastric mucus secretion and enhanced antioxidant activity of GSH, SOD and NO along with PGE_2_.

## Supporting Information

Table S1 Acute toxicity test.
(DOCX)
